# 20-Year Trends in Detection Rates of Cardia Cancer via Endoscopic Surveillance in Tianjin, China: A Hospital-Based Study

**DOI:** 10.1155/2022/1505655

**Published:** 2022-04-05

**Authors:** Rui Wang, Xiaowei Wu, Yan Song, Rui Lin, Zhongqing Zheng, Kui Jiang, Wentian Liu

**Affiliations:** Department of Gastroenterology and Hepatology, Tianjin Medical University General Hospital, Tianjin 300000, China

## Abstract

**Background:**

To analyze the time trends in cardia cancer detection rates using endoscopic surveillance from 1999 to 2019 in a high-volume Chinese hospital.

**Methods:**

In this retrospective, single-center study, data were collected from the Endoscopy Center of the Department of Gastroenterology, Tianjin Medical University General Hospital, from 1999 to 2019. Cases of cardia cancer (*n* = 1567) were extracted from a database of patients who underwent endoscopy. Clinical and epidemiological characteristics of patients with cardia cancer were analyzed, including sex, age, and proportion of early gastric cancer and degree of tumor differentiation. The joinpoint regression method was used to identify change points in incidence trends. Annual percent change (APC) values, with 95% confidence intervals (CI), were calculated for time periods before and after change points.

**Results:**

Of the 343942 patients who underwent endoscopy during 1999–2009, 1567 (4.6%) were identified with cardia cancer. The overall cardia adenocarcinoma detection rate decreased significantly from 1999 to 2004 (APC = −37.3, 95% CI: -20.9, -6.4), followed by a relatively slower decline rate from 2004 to 2019 (APC = −7.7, 95% CI: -4.4, -7.6). The crude rate of detection of early cardia cancer could not be determined by joinpoint analysis. Rates of detection reduced significantly in patients aged 60–69 and 70-79 years (APC = −8.3, 95% CI: -9.8, -6.8 and APC = −7.3, 95% CI: -8.8, -5.8, respectively). The detection rate in males decreased rapidly from 1999 to 2004 (APC = −35.9, 95% CI: -18.2, 5.6, *P* < 0.05), while the decline rate was relatively slow from 2005 to 2019 (APC = −6.9, 95% CI: -3.4, -6.1, *P* < 0.05). Among females, the detection rates also decreased from 1999 to 2004 (APC = −21.2, 95% CI: -28.1, -13.7), but remained stable from 2007 to 2019 (APC = −3.8, 95% CI: -7.9, -0.5). Detection of poorly differentiated cardia cancer also declined from 2009 to 2019 (APC = −12.8, 95% CI: -15.3, -10.0).

**Conclusions:**

The detection rate of cardia cancer among gastric cancers has been stable from 2008 to 2019. The trend of detection rate of early cardia cancer showed no significant statistical meaning; hence, it remains necessary to carefully observe the cardia area during endoscopy examination.

## 1. Background

Gastric cancer is the fifth most common malignant cancer worldwide, and the third leading cause of cancer-related death [1]. In 2018, 1,033,701 new cases and 782,685 deaths from gastric cancer were recorded globally [2, 3]. In China, gastric cancer is the second leading cause of cancer mortality [4, 5], and China is among countries with the highest burden from gastric cancer [6–10].

To reduce the socioeconomic burden related to gastric cancer, it is very important to identify individuals at high risk for gastric cancer. The strategy for early detection and diagnosis of gastric cancer can be largely divided into mass screening for the general population and surveillance for high risk individuals. Gastric cancer surveillance and diagnosis are mainly performed in medical centers, including in China and other countries that do not have universal screening strategies. Early detection of gastric cancer remains an important topic in gastroscopy, especially with regard to how the detection and diagnosis rates of early gastric cancer can be improved and the proportion of false negative diagnoses can be reduced [11]. Therefore, it is highly important to examine data from endoscopic surveillance for cardia cancer.

In the past 20 years, rapid economic growth has promoted substantial changes in lifestyles in China, alongside developments in science and technology. The detection rate of gastric cancer has also improved, due to wide availability of improved endoscopic equipment and increased levels of diagnosis and treatment in medical centers, particularly for early gastric cancer [12–14]. Therefore, it is necessary to summarize the characteristics of the diagnosis and treatment of gastric cancer in medical centers, especially cardia cancer. Description of the clinical characteristics of cardia cancer from the perspective of medical centers will assist doctors in clinical diagnosis and treatment of cardia cancer. In addition, very few studies have addressed the trends in endoscopic surveillance for cardia cancer in medical centers over time. The purpose of this study was to examine the time trends in the detection rate of cardia cancer and clinical epidemiological characteristics of patients with cardia cancer during 1999–2019 in Tianjin, China.

## 2. Methods

### 2.1. Patient Population

This was a hospital-based retrospective study. Participants were derived from the Endoscopy Center of the Department of Gastroenterology, Tianjin Medical University General Hospital, from January 1, 1999, to September 27, 2019. Gastric cancer was diagnosed following the World Health Organization diagnostic criteria for gastric cancer, based on upper gastrointestinal endoscopy and pathology [15]. According to the Siewert system, gastric cancer was classified into types I, II, and III: [16, 17] tumors with an epicenter 2–5 cm above the gastroesophageal junction (GEJ) were considered type I or distal esophageal tumors; those within 2 cm (above or below) of the GEJ were type II or true GEJ tumors; and those with an epicenter 2–5 cm distal to the GEJ were type III or subcardial tumors. Patients with type II and III tumors were included in the cardia cancer group. Exclusion criteria were the following: the diagnosis of lymphoma, neuroendocrine tumor, malignant stromal tumor, or duodenum carcinoma; gastric cancer recurrence after surgery; suspected cancer; and tumor sufficiently large to prevent origin in gastric body or cardia from being distinguished.

This study was approved by the Medical Research Ethics Committee at Tianjin Medical University General Hospital. Also, the patients were aged 22-58 years, and their underlying data were normally distributed.

### 2.2. Data Collection

Trained researchers derived the information that met the inclusion criteria from the Gastroscopy Center database, and established an EXCEL data file, with double entry and verification (Figure 1).

### 2.3. Statistical Analysis

Time trends in disease data were evaluated, and the annual percentage change (APC) in disease according to sex, age, and tumor stage was analyzed using joinpoint regression (Joinpoint Regression 2020, version 4.8.0.1, National Cancer Center). Differences with *P* < 0.05 were regarded as statistically significant.

## 3. Results

Among 343942 patients who underwent endoscopy at the Endoscopy Center, Tianjin Medical University General Hospital from 1999 to 2019, 1567 (1307 males and 260 females) diagnosed with cardia cancer were included in this study. The proportion of patients with cardia cancer among those with gastric cancer was 34.0% (1567/4610). The overall change trend in cardia cancer detection rate and the distributions of cardia and gastric cancer diagnosis rates were analyzed. Furthermore, variation in the trend of detection rates was analyzed according to various factors, including sex, age, differentiation degree, and tumor stage.

### 3.1. Trends in Detection Rates of Cardia Cancer Overall and by Tumor Stage Over Time (Tables 1 and 2 and Figures 2 and 3)

The detection rate of cardia cancer significantly decreased from 1999 to 2004 (mean APC = −37.3, 95% confidence interval [CI]: -20.9, -6.4), with a relatively slow rate of decline (APC = −7.7, 95% CI: -4.4, -7.6) from 2004 to 2019. When cardia cancer was divided into early cardia cancer and nonearly cardia cancer (referred to as advanced cardia cancer), the proportion of early cardia cancer accounted for 4.9% (77/1567). We were not allowed to make meaningful analysis for the trends of early cardia cancer due to too few cases (limited statistical power), whereas nonearly cardia cancer showed approximately the similar trends as cardia cancer overall. The proportion of cardia cancer (vs. all types of gastric cancer) detected among patients undergoing endoscopy decreased from 1999 to 2008 (APC = −3.8, 95% CI: -6.3, -1.3).

### 3.2. Trends in Detection Rates of Cardia Cancer Over Time by Sex (Table 3, Figure 4)

The rate of cardia cancer diagnosis in males decreased rapidly from 1999 to 2004 (APC = −35.9, 95% CI: -18.2, 5.6, *P* < 0.05), while the rate of decline was relatively slow from 2004 to 2019 (APC = −6.9, 95% CI: -3.4, -6.1, *P* < 0.05). Among females, diagnosis rates also decreased from 1999 to 2004 (APC = −21.2, 95% CI: -28.1, -13.7), while they remained stable from 2007 to 2019 (APC = −3.8, 95% CI: -7.9, -0.5).

### 3.3. Trends in Detection Rates of Cardia Cancer Over Time by Age (Table 4, Figure 5)

All participants were divided into five groups according to age: <50, 50–59, 60–69, 70–79, and ≥80 years old. Detection rates of cardia cancer decreased in the 60–69- and 70–79-year-old age groups (APC = −8.3, 95% CI: -9.8, -6.8 and APC = −7.3, 95% CI: -8.8, -5.8, respectively).

### 3.4. Trends in Detection Rates of Cardia Cancer Over Time by Degree of Tumor Differentiation (Figure 6, Table 5, and Table 6)

Trends in the detection rates of undifferentiated type of cardia cancer declined from 2009 to 2019 (APC = −12.8, 95% CI: -15.3, -10.0), as did those for medium and well-differentiated cardia cancer (APC = −8.4, 95% CI: -10.7, -6.1).

## 4. Discussion

This hospital-based retrospective study indicate that the detection rates of cardia cancer have decreased during the past 20 years in Tianjin, China. One of the main reasons for this finding may be that the examined population increased greatly over the study time period, with the number of included patients undergoing endoscopy in 2019 more than twenty times that in 1999. This increasing number is related to rapid economic development, leading to more patients able to afford endoscopy examination [18]. More people with low-risk of gastric cancer were undergoing endoscopy. It is one of important reasons for the declining detection rate in cardia cancer.

The proportion of cardia cancers among all types of gastric cancers showed a downward trend from 1999 to 2008 (APC = −3.8, CI: -6.3, -1.3), while there was an upward trend from 2008 to 2019 (APC = 1.2, CI: -0.5, 3.0; P = 0.1). These findings may be influenced by the overall incidence of gastric cancer, since most studies demonstrate a decreasing trend in its incidence [19, 20]. Further, there may also be a relationship with the significant decline in cardia cancer in developed areas of China in the 1990s [21, 22]. While the rate of cardia cancer compared with gastric cancer slightly increased APC = 1.2, 95% CI (-0.5, 3.0), the difference was not statistically significant. These changes may be associated with the transition towards a westernized lifestyle and increased rates of obesity in East Asia.

In our study, the overall proportion of early cardia cancer among total cardia cancer was 4.9% (77/1567). Another study reported that the proportion of early stage gastric cancers was less than 10% in China, and poor survival of patients (age-standardized 5-year relative survival, 27.4%) was observed in a population-based study from 2003 to 2005 in China [23]; however, in a report from Vietnam, the total proportion of early gastric cancer was 4.0% (115/2857). Our study provided no evidence for an increasing trend in early cardia cancer during the past two decades. It has been reported that the percentage of early cardia cancer is lower than that of early gastric cancer [24]. Further, Akashi et al. [25] reported that the cardia has looser smooth muscle bundles and more frequent large lymphatic vessels in the muscularis mucosae layer than other gastric sites, which is presumed to be one reason for the more frequent submucosal invasion in the cardia. Early detection and diagnosis of gastric cancer is difficult, because patients are asymptomatic during the early stages of the disease. The ability to detect early stage cancer during routine medical services is crucial, as it is the key to reducing gastric cancer-related mortality and improving patient survival times. Many factors can influence the diagnosis of early gastric cancer, including routine preparation before examination, type of endoscopy, use of image-enhanced endoscopy, procedure time, and alertness of endoscopists to early gastric cancer [26–28]. To reduce missed diagnoses, observation of the cardia subsite should be strengthened during endoscopic examination.

In terms of the sex differences, Holster et al. [29] reported that men are at higher risk of both cardia and noncardia gastric cancer than women. Further, Colquhoun et al. [30] reported that men had higher rates of tumor development than women at various gastric cancer subsites. The male : female ratio is approximately 3 : 1 for cardia cancer. In Sweden, Lagergren et al. reported that cardia adenocarcinoma tended to increase in young women, while the incidence of noncardia adenocarcinoma was gradually decreasing [31]. A report from India indicated that the sex ratio in gastric cancer was 1.5 : 1 in young people; however, the sex ratio increased to 3 : 1 in the population > 40 years old and to 5.6 : 1 in those >70 years old, indicating that the incidence of gastric cancer increased at a faster rate in older men than in comparable women [32]. In our study, the 60–69 and 70–79 year groups showed decreasing rates of cardia cancer detection (APC = −8.3, 95% CI: -9.8, -6.8 and APC = −7.3, 95% CI: -8.8, -5.8, respectively). Hence, the influence of age on cardia cancer incidence appears to differ according to geographical region or country. Wang et al. [1] reported that, although gastric cancer incidence rates have declined among individuals aged ≥50 years, rates are increasing among those <50 years old, particularly among women. Gastric cancer incidence declined significantly for both sexes among patients <70 years old [33].

Undifferentiated gastric cancer is less chemosensitive than other gastric cancer subtypes and an independent factor associated with poor patient prognosis and survival [34, 35]. In recent years, a decrease in the overall incidence of gastric cancer has been observed; however, the incidence of undifferentiated gastric cancer has consistently increased [36]. Our data showed declining trends in undifferentiated, as well as medium- and well-differentiated gastric cancer; however, the speed of decline in undifferentiated tumors was greater than that for medium- and well-differentiated type cancers. Many factors can influence the incidence of undifferentiated gastric cancer, potentially leading to variation among geographical regions. More effort should be focused on epidemiological analysis of undifferentiated gastric cancer.

Our study has limitations. The data were collected from a single medical center and cannot be considered sufficient to represent the true situation across the whole nation; however, Tianjin Medical University General Hospital is the largest medical center in Tianjin, which provides medical care services for more than 10 million people in the economically developed region, and thus, data from this medical center might reflect the changing trend in economically developed areas of northern China over the past 20 years. Although potential bias should be considered for different regions, the number of subjects (*n* = 343942) is sufficiently big to represent the trend across this region of China. The data in this study can represent medical service state of typical Chinese medical centers. The manual review of diagnoses conducted in this study also minimized errors, which can occur using computerized administrative coding systems.

To summarize the medical treatment and clinical practice experience can be potential to improve patient medical services. Gastric cancer represents a significant health and economic burden in many Asian countries. Early detection and treatment are significant factors that can prolong survival and reduce mortality in patients with gastric cancer. Therefore, clinicians should improve the diagnosis of early cardia cancer and focus on observation of the cardia mucosa during gastroscopy to reduce misdiagnosis. Disease trends change in response to economic growth, lifestyle changes, and advances in medical science, diagnostic methods, and treatments. Determining and developing a deep understanding of disease incidence patterns can assist in improving gastric cancer prevention strategies.

## 5. Conclusions

The detection rate of cardia cancer among gastric cancers has been stable from 2008 to 2019. Although the endoscopic equipment and technology have improved than before, the detection rate of early cardia cancer is still significantly increasing.

## Figures and Tables

**Figure 1:** 

**Figure 2:** Detection rates (per 1000 patients) of cardia cancer from 1999 to 2019 according to tumor stage.

**Figure 3:** Proportion (‰) of cardia cancer detected rate according to tumor stage.

**Figure 4:** Annual percentage change in detection rates of cardia cancer according to sex.

**Figure 5:** Annual percentage change in detection rates of cardia cancer according to age, 1999–2019.

**Figure 6:** Annual percentage change in detection rates of cardia cancer according to degree of tumor differentiation, 1999–2019.

**Table 1:** Annual percentage change in detection rates of cardia cancer and advanced cardia cancer from 1999 to 2019.

Stage	Years	APC (95% CI), ‰	*P* value
Total cardia cancer	1999–2004	-37.3 (-20.9, -6.4)	<0.05
	2004–2019	-7.7 (-4.4, -7.6)	<0.05
Advanced stage cardia cancer	1999–2004	-28.9 (-36.1, -20.8)	<0.05
	2004–2019	-7.2 (-8.7, 5.6)	<0.05

**Table 2:** Annual percentage change in proportion of cardia cancer and advanced stage cardia cancer from 1999 to 2019.

Stage	Years	APC (95% CI), %	*P* value
Advanced stage	1999–2019	-1.7 (-2.5, -0.8)	<0.05
Total cardia cancer	1999–2008	-3.8 (-6.3, -1.3)	<0.05
	2008–2019	1.2 (-0.5, 3.0)	0.1

**Table 3:** Specific change points in the trends of cardia cancer detection rate over time according to sex.

Group	Years	APC (95% CI)	*P* value
Total sample	1999–2004	-37.3 (-20.9, -6.4)	<0.05
	2004–2019	-7.7 (-4.4, -7.6)	<0.05
Female	1999–2007	-21.2 (-28.1, -13.7)	<0.05
	2007–2019	-3.8 (-7.9, -0.5)	0.1
Male	1999–2004	-35.9 (-18.2, -5.6)	<0.05
	2004–2019	-6.9 (-3.4, -6.1)	<0.05

**Table 4:** Age-group specific change points in the trends of cardia cancer detection rate over time in1999-2019.

Age (years)	APC (95% CI)	*P* value
60–69	-8.3 (-9.8, -6.8)	<0.05
70–79	-7.3 (-8.8, -5.8)	<0.05
≥ 80	-1.9 (-4.3, 0.6)	0.1

**Table 5:** Trends in detection rate of cardia cancer over time according to degree of tumor differentiation, 1999-2019.

Degree of differentiation	APC (95% CI)	*P* value
Undifferentiated	-12.8 (-15.3, -10.0)	<0.01
Medium and well differentiated	-8.4 (-10.7, -6.1)	<0.01

**Table 6:** Trends of cardia and early cardia cancer from 1999 to 2019.

Years	Population	Cardia cancer	Cardia cancer rate ‰	Early cardia cancer	Early cardia cancer rate ‰
1999	1073	30	27.96	0	0
2000	1931	54	27.97	2	1.04
2001	2275	51	22.42	0	0
2002	2563	45	17.56	0	0
2003	8228	66	8.02	0	0
2004	11891	84	7.06	2	0.17
2005	12589	85	6.75	0	0
2006	13604	86	6.32	3	0.22
2007	15476	75	4.85	0	0
2008	17097	77	4.5	0	0
2009	19298	83	4.3	3	0.16
2010	19582	89	4.55	4	0.2
2011	21937	104	4.74	3	0.14
2012	25588	92	3.6	2	0.08
2013	26841	96	3.58	2	0.07
2014	27593	95	3.44	4	0.15
2015	26256	90	3.43	8	0.31
2016	23195	74	3.19	9	0.39
2017	23028	84	3.65	16	0.7
2018	24949	58	2.33	11	0.44
2019	18634	49	2.63	8	0.43

## Data Availability

The data used and/or analyzed during the current study are available from the corresponding author on reasonable request.

## Abbreviations

CI: Confidence intervals
APC: Annual percent change
GEJ: Gastroesophageal junction.
